The article "The Change of Aqueous Humor Cytokine Levels after Anti-VEGF in Diabetic Macular Edema: A Systematic Review and Meta-Analysis" was retracted in 2023. Reasons: signs of a paper mill; suspected computer-generated content; unreliable results or conclusions; concerns about the data.

# The Change of Aqueous Humor Cytokine Levels after Anti-VEGF in Diabetic Macular Edema: A Systematic Review and Meta-Analysis

**DOI:** 10.1155/2022/9779951

**Published:** 2022-09-16

**Authors:** Aoxiang Wang, Haiyan Wang

**Affiliations:** Beijing Tongren Eye Center, Beijing Tongren Hospital, Capital Medical University, Beijing Ophthalmology & Visual Sciences Key Lab, Beijing 100730, China

## Abstract

**Background:**

Diabetic macular edema (DME) is a vision-threatening complication that severely impairs vision, and VEGF has a certain improvement effect on it as a growth factor.

**Objective:**

To assess the alterations of different aqueous humor cytokine concentrations after intravitreal antivascular endothelial growth factor (VEGF) treatment for diabetic macular edema (DME).

**Methods:**

We searched PubMed, EMBASE, and the Cochrane Library from inception up to May 2022 for studies evaluating the alterations of different aqueous humor cytokine concentrations after intravitreal anti-VEGF treatment for diabetic macular edema. The estimates from eligible studies were meta-analyzed by the Hartung–Knapp/Sidik–Jonkman random-effects method. Egger's regression test was used to determine the publications' bias. A 95% confidence interval was calculated across studies. The analysis was performed using STATA™ Version 15 software.

**Results:**

Nine eligible studies involving a total of 209 eyes for our systematic review were identified through our search strategy. The mean differences in 1-month and 2-month changes of VEGF were 110.681 pg/ml (*P* < 0.001) and 283.474 pg/ml (*P*=0.003), respectively. The mean difference in 2-month changes of interleukin 6 (IL-6) was −24.784 pg/ml (*P*=0.037). The mean difference in 3-month changes of central macular thickness was 130.372 *μ*m (*P* < 0.001).

**Conclusions:**

Intravitreal injection of anti-VEGF exerts a protective effect on macular edema secondary to diabetic retinopathy by affecting various cytokine concentrations, especially reducing aqueous VEGF concentrations and interleukin 6 in patients with DME.

## 1. Introduction

Diabetic retinopathy (DR) is a common retinal vascular disease in ophthalmology. It is a diabetic microvascular complication characterized by neovascularization. Hypoxic injury to endothelial cells leads to increased vascular permeability, mainly its early pathological changes. In the middle and late stages, retinal neovascularization and the gradual appearance of fundus proliferative membranes can eventually develop into retinal detachment, vitreous hemorrhage, and severe visual impairment. Diabetic macular edema (DME) is a sight-threatening complication that arises from the breakdown of the blood-retinal barrier (BRB) and a consequent increase in vascular permeability. Approximately 20% and 40% of patients with type 1 and type 2 diabetes mellitus, respectively, have the potential to develop into DME. One-third of patients with a diabetes mellitus duration of more than twenty years will develop DME. [1, 2].

Oxidative processes and inflammatory reactions have been considered significant procedures in the pathogenesis of DME, which lead to the upregulation of multiple cytokines and growth factors. [3, 4] The overexpression of these molecules, including vascular endothelial growth factor (VEGF), angiopoietins, tumor necrosis factor (TNF), monocyte chemoattractant protein (MCP), and so on, is responsible for the dysfunction of BRB and the development of DME. [4].

Tremendous progress has been made in the treatment of DME in recent years. Especially, the recognition of VEGF as the potent regulator to cause vascular leakage has led to the development of VEGF-inhibiting drugs. Anti-VEGF therapy has become the initial treatment option for patients with macular edema secondary to DR. Several anti-VEGF drugs target the VEGF molecule and have slightly different action mechanisms. Ranibizumab is a monoclonal antibody that blocks all isoforms of VEGF-A. Bevacizumab is a full-length humanized monoclonal antibody and blocks all isoforms of VEGF-A. Aﬂibercept is a soluble protein that contains extracellular VEGF receptor 1 and 2 sequences fused to the Fc domain of a human immunoglobulin-G1 molecule and blocks all isoforms of VEGF [4]. Besides steroids and nonsteroids, anti-inﬂammatory drugs are also widely used in the clinic because of the important role of inflammation in the pathogenesis of DME. Visual acuity improvement after intravitreal dexamethasone has been confirmed in the previous study [5].

A variety of studies concerning the change of aqueous humor cytokine levels in patients with macular edema caused by DR have been submitted. Despite the growing evidence of clear results, systematic and comprehensive evaluations of cytokine levels after anti-VEGF to treat DME have yet to be published. Therefore, we undertook a meta-analysis of multiple cytokines in aqueous humor to assess the change in those after anti-VEGF intravitreal injection in patients with DME.

## 2. Methods

### 2.1. Search and Identiﬁcation Strategy

We conducted searches of PubMed, EMBASE, and the Cochrane Library from their inception until May 1, 2022, using the terms *diabetic macular edema or DM* and *bevacizumab, ranibizumab, aflibercept, conbercept, anti-VEGF agents,* and *aqueous humor cytokine*. Language or study-design restrictions were not used. When titles and/or abstracts fit our search terms, the abstracts were reviewed to exclude irrelevant studies (e.g., case reports, reviews, or experimental treatments). We then carefully read all the remaining articles to determine whether they contained data that was applicable to our study.

### 2.2. Inclusion and Exclusion Criteria

The studies were included in the meta-analysis if they fulfilled the following criteria [1]: all observational studies investigating the change of aqueous humor cytokine levels after anti-VEGF treatment in patients with DME [2]; data of aqueous humor cytokine levels pretherapy and post-treatment were reported [3]; all measured data were reported as mean/mean difference and standard deviation. The studies where the mean difference could be calculated indirectly from the data provided in the study were considered eligible for inclusion in our meta-analysis.

We excluded conference abstracts, letters to the editor, case-report studies, systematic reviews, meta-analyses, nonhuman studies, and full texts without raw data for retrieval (a detailed analysis of this study is not possible without the original data).

### 2.3. Data Extraction and Quality Assessment

The following information on study characteristics and clinical treatments was collected from all included studies: publication metrics (name of the first author), year of publication, location of study, subject information (age, gender, and length of follow-up period), treatment information (applied treatment, injection frequency, and number of subjects in each interventional group), and outcomes at a specific time, including VEGF, interleukin 6 (IL-6), interleukin 8 (IL-8), inducible protein 10 (IP-10), MCP-1, and central macular thickness (CMT). The two authors independently extracted the data from each of these studies using the standardized data extraction format prepared in a Microsoft™Excel worksheet. The two investigators mentioned above assessed the methodologic quality of included studies through a modiﬁed version of the Newcastle-Ottawa Scale (NOS) for cohort studies [6]. The NOS was used to assess the risk of bias of the studies by analyzing the following eight items: representativeness of the exposed cohort, selection of nonexposed cohort, ascertainment of exposure, the outcome of the interest declared at the start of the study, comparability of a cohort, assessment of outcome, follow-up duration, and adequacy of follow-up of cohorts [6]. All eligible studies were of moderate or high quality (scored ≥6).

### 2.4. Statistical Analysis

Means and standard deviations from each outcome group were used to calculate weighted mean differences (WMDs) of each cytokine measurement between different outcome groups, with corresponding 95% confidence intervals (95% CI). In cases where values of cytokine measurement outcomes were not directly available, for example, some studies reported the value using the median, the minimum, and maximum values, and/or the first and third quartiles. We transformed those data into the mean and standard deviation by adopting the Dehui Luo and Xiang Wan method [7, 8]. If there were two subgroups (such as responders and nonresponders) in one study, we used the following formula to combine the two groups into one intervention group [9]:

(1) $$\begin{array}{c} \text{combined }S\;D=\sqrt{\frac{\left(N_{1}-1\right)SD_{1}^{2}+\left(N_{2}-1\right)SD_{2}^{2}+\left(N_{1}N_{2}/N_{1}+N_{2}\;\right)\left(\left(M_{1}^{2}+M_{2}^{2}-2M_{1}M_{2}\right)\right)}{N_{1}+N_{2}-1}.} \end{array}$$

Where *N* = sample size and *M* = mean.

We analyzed the quantitative evidence with Stata 15.0 software for Mac. Continuous data were expressed as means and standard deviations and WMD were calculated. Cochran's *Q* chisquare statistics and I^2^ statistical tests were conducted to assess the random variations in primary studies [10]. Herein, *P* < 0.1 and I^2^ ≥ 50% indicated considerable heterogeneity. Random effect models were used to pool the data since the interventions varied among the included studies. Potential publication bias was assessed by visually inspecting funnel plots and objectively using the Egger bias test with *P* > 0.05, indicating negative publication bias. A sensitivity analysis was used to see the effect of a single study on the overall effect estimation. *P* values less than 0.05 were defined as significant.

### 2.5. Presentation and Reporting of Results

The results of this review were reported based on the Preferred Reporting Items for Systematic Review and Meta-Analyses (PRISMA) statement guidelines [11]. The entire process of study screening, selection, and inclusion was described with a flow diagram. The results were presented using forest plots and summary tables.

## 3. Results

### 3.1. Baseline Characteristics of Included Studies

We identified 83 publications by the search terms prior to August 2021. After the removal of duplicates, 23 articles were selected for the title and abstract screening, and 5 of them were excluded. The remaining 18 articles were eligible for full-text review. We excluded nine articles since one of them was not available, and eight articles did not include eligible measurements. Thus, nine prospective studies were included in our systematic review and were eligible for meta-analysis [12–19] (Table 1). The literature selection process and reasons for exclusion are summarized in (Figure 1).

Overall, sample sizes varied from 9 to 48 eyes, with a total of 209 eyes included in the analyses, and the duration of follow-up time ranged from 1 to 2 months. The study (ETDRS) letter scores or Snellen acuity fraction were transposed to the logarithm of the minimum angle of resolution (log MAR) units [20]. The mean age ranged from 54.45 to 69.25 years, and the mean baseline BCVA logMAR scores and CMT ranged from 387.7 to 570.0 *μ*m, respectively. There were 5 studies treated with ranibizumab, 2 studies with aflibercept, and 1 with bevacizumab. All eyes received monthly anti-VEGF injection monotherapy in nine studies. To unify this meta-analysis, the selected cytokines in our study were VEGF, IL-6, IL-8, IP-10, and MCP-1 (pm/ml). See Table 2.

### 3.2. VEGF Level Declined in the Two-Month following after Treatment

The VEGF level of each study from baseline to different follow-up times. One-month following intravitreal treatment, VEGF levels in 53 eyes across three studies declined with a mean of 110.68 pg/ml (95% CI: −163.581 to −57.782 pg/ml, *P*=0.203, I2=37.2%; figure 2(a)). Two-month following the treatment, VEGF of 169 eyes in five studies with a mean reduction of 283.47 pg/ml (95% CI: −470.40 to 96.54 pg/ml, *P* < 0.001, I2=97.0%; Figure 2(b)). The evidence from Egger's test showed no significant proof of publication bias (*P*=0.07).

### 3.3. The IL-6 Level Was Downregulated in One-Month and Two-Month following after Treatment

Four types of research showed IL-6 levels after one-month following the treatment. The IL-6 level was obviously decreased 1 month after treatment (mean level=−16.569 pg/ml, 95% CI: −40.36 to 7.22 pg/ml, *P*=0.029, I^2^=66.7%) and the evidence showed no significant proof of publication bias that was showed after Egger's test (*P*=0.99). While a mean reduction of −24.78 pg/ml could be found at the 2-month time point (95% CI: −48.13 to −1.43 pg/ml, *P*=0.002, I^2^=73.6%). Sensitivity analysis did not show the effect of a single study on the overall effect estimation as shown in Figure 3.

### 3.4. The Mean Change of MCP-1, IL-8, and IP-10 in the Posttreatment

There was no signiﬁcant difference between baseline and posttreatment (including month 1 and month 2) during the mean change of MCP-1(MCP-1 : WMD=−215.18 pg/ml, 95% CI: −599.72 to 169.35 pg/ml, *P*=0.985, I^2^=0.0%; WMD=−102.49 pg/ml, 95% CI: −235.57 to 30.59 pg/ml, *P*=0.192, I^2^ = 32.5%) and IP-10 (WMD=22.54 pg/ml, 95%CI: −55.72 to 100.80 pg/ml, *P*=0.337, I^2^=11.1%; WMD=29.44 pg/ml, 95% CI: −73.66 to 132.54 pg/ml, *P*=0.088, I^2^=58.8%, Egger's test: *P*=0.633). On the other hand, no alteration of the level of IL-8 was found in the one-month following treatment (WMD=1.85 pg/ml, 95% CI: −5.39 to 9.08 pg/ml, *P*=0.931, I^2^=0.0%); however, a mild drop appeared after two months of treatment (WMD=−0.31 pg/ml, 95% CI: −4.03 to 3.41 pg/ml, *P*=0.045, I^2^=55.9%, Egger's test: *P*=0.55). The details are shown in Table 3, Figures 4 and 5.

### 3.5. Central Macular Thickness

Among the nine studies, three recorded the CMT change at the three-month follow-up time. We found a mean thickness of CMT (130.37 *μ*m) of 106 eyes (95% CI: −163.72 to −97.02 *μ*m, *P*=0.388, I^2^=0.0%). The result is displayed in Figure 6.

## 4. Discussion

Diabetic macular edema is the most common manifestation of DR, which can cause vision impairment in patients with diabetes [19]. In addition, many intraocular cytokines have been involved in the development of DME, which have been reported to demonstrate the severity of DME and have been found to positively correlate with the CMT and cytokine levels [14]. In this meta-analysis, we examined nine studies representing 209 eyes based on a robust search method and precise data extraction following a systematic review process. Based on the studies enrolled in this meta-analysis, most articles reported obvious alterations in VEGF and IL-6, which were consistent with our overall results. Our analysis showed synthesized evidence on the change of different aqueous humor cytokine levels in patients with DME globally. Due to the limited data, it was impossible to evaluate treatment efficacy at longer time points.

Based on the pooled data analysis, VEGF significantly decreased at 1 month and 2 months after anti-VEGF treatment, and the decline of IL-6 and IL-8 can be observed at the 2-month follow-up point. The statistical differences were not demonstrated in the alterations of MCP-1 and IP-10 during the follow-up period. In addition, CMT significantly decreased after two monthly intravitreal anti-VEGF injections.

VEGF is a dominant proangiogenic factor and increases microvascular permeability. Vitreous or aqueous levels of VEGF are reportedly related to retinal vascular permeability and the severity of DME. Also, injections of anti-VEGF reagents have become the first-line treatment worldwide in DME patients [21]. Notably, our results demonstrated a decrease in VEGF and CMT. This was evident, which proved the validity of the anti-VEGF treatment during the follow-up time. Our results have demonstrated the statistically significant relationship between eyes with DME undergoing anti-VEGF therapy and lower aqueous humor VEGF concentration early in treatment. Although there was a considerably lower concentration of VEGF in all eyes following two months of anti-VEGF treatment, the 2-month follow-up VEGF concentration was remarkably downregulated compared to that of the baseline.

Some secreted cytokines and growth factors are activated and involved in the procedure of the BRB alteration [20]. IL-6 is an inflammatory cytokine involved in the enhancement of vascular permeability and the alterations of BRB in DME. The level of VEGF has been reported to be strongly correlated with IL-6 concentration in aqueous humor and vitreous, although it has not been found to have any close association between IL-6 and the severity of DME (22). Our results showed that at the 1-month follow-up, the decline was not observed. At the 2-month follow-up, there was a significant decrease in IL-6. Whereas, IL-8 is a main activator and attractant of neutrophils and T lymphocytes and is reported to be related to proliferative DR and related to the IL-8 level change in the aqueous humor which may be difficult to observe in the short term [22, 23]. At the 2-month follow-up, a mild drop in IL-8 level was discovered in our results. Moreover, a previous study has indicated that IL-8 may be a representative marker of chronicity in DR [24]. Therefore, the upregulation of IL-8 may remain for a long time in the aqueous humor.

IP-10 is a cytokine that can enhance immune reactivity but is a potent inhibitor of both IL-8- and FGF-induced angiogenic activity. MCP-1 induces monocyte and macrophage inﬁltration into tissues without activating neutrophils. A previous study found that IP-10 and MCP-1 were much higher in severe nonproliferative diabetic retinopathy and proliferative DR than in less severe DR (26). In addition, Hideharu and his colleagues [25] found that MCP-1 played a relatively less important role than VEGF in DR and DME. These findings may explain why the great changes in MCP-1 and IL-8 cannot be observed in chronic inflammation without a long course of DR.

This study still has a few limitations. First, some cytokines in DME eyes were reported to decrease compared to healthy eyes in previous cross-section studies, but the trends of decline were not found in our results of 2-month follow-up in comparison with the baseline [12, 18, 22, 25–27]. In addition, more kinds of cytokines should be recruited for further analysis. At last, the efficacy of the change may be related to the category of anti-VEGF drugs. For example, study [14] found that ranibizumab could have a more potent effect on the profile of the intraocular cytokine than bevacizumab. Consequently, a larger sample size and long-term studies are required to investigate changes in different cytokines in aqueous patients suffering from DME and better understand the timing of therapy efficacy for clinics.

## 5. Conclusion

This study aimed to provide new insights into changes in aqueous humor cytokines following anti-VEGF intravitreal injections in DME. Our results have presented positive evidence for the change of different aqueous cytokine levels after anti-VEGF treatment in patients with DME. These findings may lead to further understanding of the disease process and aid future treatment strategies. Even so, more long-term data are needed to improve this meta-analysis accuracy and provide clinical guidance.

## Figures and Tables

**Figure 1:** The flow diagram of the literature selective process and reasons for exclusion.

**Figure 2:** (a) VEGF of 53 eyes in three studies in one month following the intravitreal treatment; (b) VEGF of 169 eyes in five studies in two-month following the intravitreal treatment.

**Figure 3:** (a) The level of IL-6 in four studies of one-month following the treatment; (b) IL-6 level in six studies of two-month following the treatment.

**Figure 4:** The mean change of IL-8, IP-10, and MCP-1 after 1-month treatment.

**Figure 5:** The mean change of IL-8, IP-10, and MCP-1 after two-month treatment.

**Figure 6:** The change in the CMT at the three-month follow-up time.

**Table 1:** Nine studies were included in our systematic review and were eligible for meta-analysis.

Study	Selection				Comparability	Exposure			
	Represent	Selection	Ascertain	Demon	Comparability of cohorts	Assessment of outcome	Follow-up long enough for outcomes	Adequacy of follow-up	Scores
Japan, Takuya utsumi	☆	☆	☆	—	☆	☆	—	☆	6
Japan, Tomoyasu	☆	☆	☆	—	☆	☆	—	☆	6
Austria, Dominika	☆	☆	☆	—	☆☆	☆	☆	☆	8
Italy, Mastropasqua	☆	☆	☆	—	☆☆	☆	☆	☆	8
Canada, Verena	☆	☆	☆	—	☆	☆	—	☆	6
Canada, Tina	☆	☆	☆	—	☆	☆	—	☆	6
Australia, Shueh	☆	☆	☆	—	☆	☆	—	☆	6
Canada, Roxane	☆	☆	☆	—	☆	☆	—	☆	6
Korea, Hee Jin Sohn	☆	☆	☆	—	☆☆	☆	—	☆	7

Note. represent, representativeness; ascertain, ascertainment; demon, demonstration.

**Table 2:** Study characteristics of the nine trials in the meta-analysis.

Country, author, year	Study design	Treatment	S.S	Age (y) (Mean ± SD)	Baseline CFT (*μ*m)	Baseline BCVA, logMAR	Cytokine recorded in our meta-analysis	Follow-up month
Japan, Takuya et al., 2021	Self-control (prospective)	Ranibizumab	25	62.9 ± 9.6	560 ± 166	0.51 ± 0.30	VEGF, IL-6, IL-8, IP-10, and MCP-1	1
Austria, Dominika et al., 2020	Self-control (prospective)	Ranibizumab and dexamethasone	9	66.9 ± 8.8; 64.6 ± 9.0^*∗*^	440 ± 144; 471.3 ± 122.6^*∗*^	0.70; 0.35^*∗*^	VEGF, IL-6, IL-8, and MCP-1	2
Canada, Verena et al., 2020	Self-control (prospective)	Aﬂibercept	17	57.2 ± 8.1	430.9 ± 85.5	0.39 ± 0.16	VEGF, IL-6, IL-8, IP-10, and MCP-1	1 and 2
Canada, Tina et al., 2019	Self-control (prospective)	Ranibizumab	35	62.4 ± 7.3	480.4 ± 117.4	0.60 ± 0.30	VEGF, IL-6, IL-8, and MCP-1	2
Italy, Mastropasqua et al., 2018	Self-control (prospective)	Aflibercept	20	63.4 ± 7.3	469.43 ± 181.91	0.46 ± 0.24	VEGF, IL-6, IL-8, IP-10, and MCP-1	2
Australia, Shueh et al., 2018	Self-control (prospective)	Ranibizumab	25	63.8 ± 9.6	484.5 ± 134.3	0.48 ± 0.20	IL-6, IL-8, IP-10, MCP-1	2
Canada, Roxane et al., 2018	Self-control (prospective)	Ranibizumab	48	61.9 ± 7.1	495.0 ± 134.6	0.60 ± 0.30	VEGF, IL-6, IL-8, and MCP-1	2
Japan, Tomoyasu et al., 2017	Self-control (prospective)	Ranibizumab	13	62.5 ± 11.9	570.0 ± 109.8	0.47 ± 0.25	IL-6, IL-8, IP-10, and MCP-1	1
Korea, Hee Jin Sohn et al., 2011	Self-control (prospective)	Bevacizumab	11	54.4 ± 10.2	387.7 ± 111.3	0.44 ± 0.32	VEGF, IL-6, IL-8, IP-10, and MCP-1	1

Note. S.S, sample size; ^*∗*^the BCVA of two groups in the original text was 74.78 ± 14.85 and 67.22 ± 10.52 presented by Early Treatment Diabetic Retinopathy Study (ETDRS) letter scores. The SD was not available due to lack of raw data.

**Table 3:** The mean changes of MCP-1, IL-8, and IP-10 after treatment.

Index	WMD (95%CI) pg/ml	I^2^ (%)	*P*
After one-month treatment			
MCP	−215.18(−599.72,169.35)	0.0	0.985
IL-8	1.85(−5.39,9.08)	0.0	0.931
IP-10	22.54(−55.72,100.80)	11.1	0.337

After two-month treatment			
MCP	−102.49(−235.57,30.59)	32.5	0.192
IL-8	−0.31(−4.03,3.41)	55.9	0.045^*∗*^
IP-10	29.44(−73.66,132.54)	58.8	0.088

Note. WMD, weighted mean difference; ^*∗*^*P* < 0.05.

## Data Availability

The datasets used and analyzed during the present study are available from the corresponding author upon reasonable request.
